The article "Honokiol Inhibits Proliferation, Invasion and Induces Apoptosis Through Targeting Lyn Kinase in Human Lung Adenocarcinoma Cells" was published in 2018. Journal: Front Pharmacol.

# Honokiol Inhibits Proliferation, Invasion and Induces Apoptosis Through Targeting Lyn Kinase in Human Lung Adenocarcinoma Cells

**DOI:** 10.3389/fphar.2018.00558

**Published:** 2018-05-28

**Authors:** Xi Dai, Run-Ze Li, Ze-Bo Jiang, Chun-Li Wei, Lian-Xiang Luo, Xiao-Jun Yao, Guo-Ping Li, Elaine L.-H. Leung

**Affiliations:** ^1^State Key Laboratory of Quality Research in Chinese Medicines, Macau Institute for Applied Research in Medicine and Health, Macau University of Science and Technology, Macau, China; ^2^Department of Respiratory Medicine, Affiliated Hospital of Southwest Medical University, Luzhou, China; ^3^Department of Respiratory Medicine, The Third People’s Hospital of Chengdu, The Affiliated Hospital of Southwest Jiaotong University, Chengdu, China

**Keywords:** honokiol, Lyn kinase, EGFR, apoptosis, Lung cancer

## Abstract

Honokiol is a natural compound with small molecular structure and extracted from bark of magnolia trees. The biological activities of honokiol include anti-oxidation, anti-inflammation as well as anti-tumor. However, their mechanism remains unknown. In this study, A549 cell line and EGFR-mutant cell line PC-9 with higher expression level of Lyn than A549 cells were used to assess the anti-tumor effects of honokiol. As shown in this study, honokiol is an effective drug on inhibiting proliferation and inducing apoptosis depended on Lyn and EGFR signal pathway regulated by Lyn, and its efficacy is stronger in PC-9 cells than A549 cells. In addition, this anti-tumor effect in PC-9 cells was weakened by Lyn-knockdown. Taken together, this study indicated the mechanism of honokiol on lung adenocarcinoma and provides a possibility of honokiol as an effective anti-tumor medicine.

## Introduction

Lung cancer is the most prevalent type of cancer as well as the most common cause of death from cancer worldwide (Siegel et al., 2013). According to a global statistic on lung cancer, there are more than 1.825 million new case and 1.59 million deaths every year, and more than 55% of the world’s lung cancer cases occur in Asia. In both China and the United States, lung cancer is the most common incident cancer and the leading cause of cancer death (Siegel et al., 2016), and cause huge mortality to population. Recently, targeting therapy, such as EGFR tyrosine kinase inhibitors (TKIs) or VEGF receptor inhibitors, improve response rates, time to progression, and overall survival. Unfortunately, only about 10% patients with EGFR mutant benefit from TKI and most of them develop disease progression after a median of 9.2–14.7 months of TKI therapy. Acquired resistance caused by T790M mutation remains a significant barrier to effective treatment referred to patients with EGFR-mutant NSCLC (Westover et al., 2018; Wu and Shih, 2018). Additionally, these therapies lead to side effects which bring pain to patients. Therefore, novel and effective preventive and therapeutic agents should be developed to combat this major health problem.

Traditional Chinese medicine (TCM) for cancer treatment has more than 2000 years history. Concepts of diagnosis and treatment methods in TCM demonstrate characteristics and advantages of TCM-based herbal medicines and laid the foundation or the innovation and development of cancer treatment with TCM (Liu et al., 2015). Obviously, TCM contains various natural compounds which are the most prolific source of leading compounds for drug development. Usually, TCM has therapeutic efficacy in lung cancer with various biological activity and minimal side effects. For these reasons, TCM has gained increasing interest and acceptance worldwide, especially TCM-based herbal drugs that selectively target molecular pathways in cancer cells and modulates proliferation and progression of cancer. On the other hand, current clinical systemic treatments for NSCLC is low efficacy but high toxicity. TCM-based herbal medicines may increase efficacy of chemotherapy (McCulloch et al., 2006).

Honokiol is a natural compound isolated from the bark and root of Magnolia officinalis and used as traditional Chinese herbal medicine for thousands of years for the treatment of various diseases. The biological activities of honokiol includes anti-oxidative, anti-allergic, anti-inflammatory, anti-bacterial, and many previous studies have indicated that honokiol is a useful biologically active compound in protecting against hepatotoxicity, neurotoxicity, thrombosis and angiopathy (Fried and Arbiser, 2009). Recently, the anti-cancer activities of honokiol have gained increasing number of attention and various mechanisms have been reported (Bai et al., 2003; Chen et al., 2004; Battle et al., 2005; Jiang et al., 2008; Park et al., 2009). However, the mechanisms of antitumor activity of honokiol are still unclear completely. In this present study, we used A549 cell line and EGFR-mutant cell line PC-9 with higher expression level of Lyn than A549 cell line to clarify the *in vitro* antitumor effects and treatment mechanism of honokiol.

## Results

### Honokiol Inhibits Cell Proliferation in Both A549 Cells and PC-9 Cells

As shown in **Figure 1B**, compared with A549 cells which harbors EGFR wild type, the expression level and activity of Lyn were markedly increased as well as the expression level and activity of EGFR in PC-9 cells with EGFR mutation. MTT assay was used to assess the cytotoxicity of honokiol on A549 cells and PC-9 cells. Honokiol was tested in both cell lines for 24, 48, and 72 h at an increasing concentration of 0, 20, 40, 60, and 80 μM. The percentage of cell viability and the IC_50_ values were analyzed with GraphPad Prism 5.0 software. As shown in **Figure 1A**, honokiol inhibited the proliferation rate of PC-9 cells in a concentration dependent and time-dependent manner. In addition, honokiol showed lower cytotoxicity in A549 cells than PC-9 cells. The IC_50_ value of PC-9 cells at 24, 48, and 72 h were all lower than that of A549 cells. This result implied that honokiol has stronger cytotoxic effect on PC-9 cells with higher expression level of Lyn kinase (**Figure 1B**).

**FIGURE 1:** Effects of honokiol on cell viability in A549 cells and PC-9 cells. **(A)** The percentage of cell viability of PC-9 cells treated with various concentration of honokiol (0, 20, 40, 60, and 80 μM) for 24, 48, and 72 h, and a comparison of cell viability and IC_50_ between A549 cells and PC-9 cells at different exposing time in honokiol. **(B)** A comparison of expression level of Lyn and EGFR between A549 cells and PC-9 cells, as analyzed by Western blots assay. ^∗∗^*P* < 0.05 and ^∗∗∗^*P* < 0.01 for comparison between two groups.

### Honokiol Inhibits Colony Formation and Invasion in PC-9 Cells

Honokiol was an effective drug to modulate cell proliferation. As same as the results of MTT assay, honokiol significantly inhibited the colony formation capacity in PC-9 cells in a concentration dependent manner (**Figure 2A**). Moreover, the wound healing assay and transwell invasion assay were used to evaluate the impact of honokiol on cell migration and invasion. Consistent with previous finding from MTT assay and colony formation assay, we also found that honokiol significantly inhibited the migration and invasion capacity of PC-9 cells (**Figures 2B,C**).

**FIGURE 2:** Effects of honokiol on colony formation, migration, and invasion in PC-9 cells. **(A)** Colony formation of PC-9 cells treated with various concentration of honokiol (0, 20, 40, 60, and 80 μM) for 10 days was assessed. **(B)** Migration of PC-9 cells treated with various concentration of honokiol into wound was assessed at 0, 12, and 24 h post scratch. **(C)** Invasion of PC-9 cells treated with various concentration of honokiol was assessed for 24 h. ^∗^*P* > 0.05, ^∗∗^*P* < 0.05 and ^∗∗∗^*P* < 0.01 for comparison among groups.

### Honokiol Induces Apoptosis in PC-9 Cells

Flow cytometry was used to analyze the percentage of apoptosis cells after treated with honokiol. Our results showed that honokiol induced apoptosis in PC-9 cells in a concentration dependent manner. Images picked from microscope at 40× magnification also showed deformation, death and floating of PC-9 cells induced by honokiol (**Figures 3A,B**).

**FIGURE 3:** Honokiol induced apoptosis and down-regulated Lyn and Lyn-mediated EGFR signaling in PC-9 cells. **(A)** Apoptosis of PC-9 cells treated with various concentration of honokiol for 24 h was analyzed by flow cytometer. **(B)** Representative pictures of PC-9 cells treated with various concentration of honokiol for 24 h were picked with microscope (40×). **(C)** Lyn, p-Lyn, EGFR, p-EGFR, PI3K, p-PI3K, AKT, p-AKT, STAT3, and p-STAT3 protein expression of PC-9 cells were detected by Western blots assay after treated with honokiol (0, 20, 40, and 60 μM) for 24 h. The non-specific Src tyrosine kinase inhibitor (TKI) PP2 is the positive control. ^∗^P > 0.05 and ^∗∗∗^P < 0.01 for comparison among groups.

### Honokiol Suppresses Lyn Kinase and EGFR Signaling Pathway in PC-9 Cells

PC-9 cell line is one of the EGFR mutation cell line with continuous activation of EGFR. In our previous study, we have found Lyn was an effective regulator on EGFR signaling pathway, therefore, we detected the effect of honokiol on Lyn and it mediated EGFR signaling transduction in PC-9 cells. PP2 is a non-specific Src TKIs, as a positive control in this study.

As shown in **Figure 3C**, honokiol decreased the expression level of Lyn and its phosphorylation status significantly. In addition, treatment with honokiol also led to a reduction of EGFR/PI3K/AKT and STAT3, and their phosphorylation status. These results indicated that honokiol inhibits PC-9 cell proliferation, invasion and induces apoptosis through targeting Lyn kinase and Lyn-mediated EGFR signaling pathway.

### Lyn Kinase Is Critical for Honokiol Inhibiting Proliferation, Invasion and Inducing Apoptosis in PC-9 Cells

To further evaluate the role of Lyn kinase for the effects of honokiol, PC-9 cells were transfected with Lyn small interfering RNA (Lyn-siRNA) for Lyn knockdown. The expression level of Lyn kinase was analyzed by Western blots analysis. **Figure 4A** showed the expression level of Lyn and p-Lyn were decreased significantly after administration with Lyn-siRNA. Based on this, MTT assay was used to assess the cytotoxicity of honokiol on PC-9 cells with or without Lyn siRNA knockdown. As shown in **Figure 4B**, the cytotoxicity of honokiol at a concentration of 60 μM for 24, 48, and 72 h were all weakened by Lyn knockdown. More than this, the wound healing assay and transwell invasion assay also indicated that the inhibition effects of honokiol at a concentration of 60 μM on migration and invasion capacity of PC-9 were weakened by Lyn knockdown (**Figures 4C–F**). Additionally, Western blots analysis was used to detect the protein expression of EGFR/PI3K/AKT and STAT3 in Lyn-knockdown PC-9 cells after treatment with honokiol. As shown in **Figure 5A**, the expression levels of EGFR, PI3K, AKT, STAT3 and their phosphorylation status were higher in honokiol-induced Lyn-siRNA transfected PC-9 cells than in control cells. This result proved that Lyn played an important role for honokiol. Taken together, honokiol is an effective TCM to inhibit lung cancer growth through targeting Lyn kinase.

**FIGURE 4:** Inhibition effects of honokiol on cell proliferation, migration and invasion of PC-9 cells was weakened by Lyn-knockdown. **(A)** Lyn and p-Lyn protein expression in wide type PC-9 cells and Lyn-knockdown PC-9 cells were detected by Western blots assay. **(B)** The percentage of cell viability of PC-9 cells with or without Lyn-siRNA transfection at 60 μM concentration of honokiol for 24, 48, and 72h. **(C,E)** Migration of PC-9 cells with or without Lyn-siRNA transfection into wound was assessed at 0h, 12 and 24 h post scratch at 60 μM concentration of honokiol. **(D,F)** Invasion of PC-9 cells with or without Lyn-siRNA transfection was assessed for 24 h at 60 μM concentration of honokiol. ^∗^P > 0.05, ^∗∗^P < 0.05 and ^∗∗∗^P < 0.01 for comparison among groups.

**FIGURE 5:** Effect of honokiol on down regulation of EGFR signaling in PC-9 cells was weakened by Lyn knockdown. **(A)** EGFR, p-EGFR, PI3K, p-PI3K, AKT, p-AKT, STAT3, and p-STAT3 protein expression in wide type PC-9 cells and Lyn-knockdown PC-9 cells were detected by Western blots assay after treated with honokiol (60 μM) for 24 h. **(B)** Graphical abstract showed the antitumor mechanism of honokiol on lung adenocarcinoma. ^∗^P > 0.05, ^∗∗^P < 0.05 and ^∗∗∗^P < 0.01 for comparison among groups.

## Discussion

Several studies on honokiol have suggested that it has multiple mechanisms of antitumor properties such as anti-tumor growth, anti-migration, anti-angiogenesis, or overcoming multiple drug resistance (MDR) (Kumar et al., 2013). Honokiol induces apoptosis in chronic lymphocytic leukemia cells through activation of Caspase-8 and Bax, it also potentiates the cytotoxicity of anti-leukemia chemotherapeutic drugs (Battle et al., 2005). Additionally, subsequent reports also found honokiol induced apoptosis on colon cancer and breast cancer. Honokiol prevents the growth of RKO cells and MDA-MD-231 cells through targeting p53 and KRAS signaling (Wang et al., 2004; Wolf et al., 2007). Of interest, honokiol was also observed to induce apoptosis through increasing the expression of Bax, while decreasing the expression of Bcl-2 in KRAS-mutant lung cancer cells (Luo et al., 2017). Moreover, one study suggests that cyclophilin-D is likely a target of the cytotoxic action of honokiol (Li et al., 2007). In this research, cells from high-grade esophageal dysplasia were found to highly sensitive to honokiol, but this sensitivity could be weakened by cyclophilin-D siRNA. On the other hand, honokiol has been shown to overcome MDR during cancer progression. In a nude mice xenograft model research, in combination with honokiol, docetaxel showed a reduction in tumor volume as well as microvessel count in nude mice significantly (Shigemura et al., 2007), combination of honokiol with DDP enhancing the treatment efficacy of lung cancer as well (Jiang et al., 2008). Subsequent study demonstrated that honokiol modulated MDR due to down-regulated NF-κB signaling (Ahn et al., 2006). Honokiol has efficacy to enhance the activation of TNF-α, in this way, honokiol inhibits activation of NF-κB and Akt. As a result, honokiol dramatically decreases expression level of NF-κB target genes, such as VEGF, MMP-9, and COX-2. In summary, honokiol is an effective antitumor agent due to its multiple function effects and multiple signaling pathways undergoing its regulation.

EGFR over-expression and mutation have been demonstrated as an important factor for growth and progression of lung adenocarcinoma (Merrick et al., 2006), but treatment efficacies of EGFR TKIs are weak and limited due to TKIs-related toxicities or high risk in part of patients (Rosenthal et al., 2014). Therefore, it’s prudent to develop effective and safe drugs targeting EGFR in lung adenocarcinoma. A little part of previous reports indicated honokiol regulated EGFR and its downstream effectors. Song’s research indicated that honokiol decrease the expression of EGFR and its downstream effective proteins (Song et al., 2016). Lee also reported magnolol inhibits EGFR-mediated signaling pathways in prostate cancer (Lee et al., 2009). In addition, honokiol was reported to enhance the efficacy of EGFR TKIs (Leeman-Neill et al., 2010).

Lyn is a member of the Src family of non-receptor tyrosine kinase and an important regulator of immune homeostasis and pattern recognition receptor-induced responses. Src kinase family has been reported playing an important role in VEGF signaling and effecting proliferation and migration of cancer cell, and Yes and Lyn kinase were highly associated with EGFR signaling (Munshi et al., 2000; Iida et al., 2013). Previous studies reported that EGFR promotes DNA replication of cancer cell by Lyn phosphorylation, and Lyn kinase regulates phosphorylation of EGFR through PKCβII (Huang et al., 2013; Sutton et al., 2013). In our previous research, Lyn kinase was demonstrated to be an important factor up-regulating activity of EGFR and its downstream signaling pathway by phosphorylating tyrosine 845 of EGFR which suggests the therapeutic target for lung adenocarcinoma. Here, honokiol has stronger cytotoxic effect on PC-9 cells with higher expression level of Lyn kinase than A549 cells in this study, and honokiol decreased expression level of Lyn significantly in a dose-dependent manner. Moreover, after Lyn silencing, the regulating effect of honokiol on EGFR and its downstream effectors were weakened. Taken together, we reported for the first time that honokiol inhibits EGFR and its downstream signaling pathway by targeting Lyn kinase (**Figure 5B**).

## Materials and Methods

### Cell Culture and Reagents

A549 cells and PC-9 cells were obtained from American Type Culture Collection (ATCC) and cultured at 37°C in a humidified atmosphere of 5% CO2 with RPMI-1640 medium, which supplemented with 10% fetal bovine serum (FBS), 100 units/ml penicillin and 100 μg/ml streptomycin. Honokiol reagent was purchased from Selleck Chemicals. The primary antibodies of Lyn, p-Lyn, EGFR, p-EGFR, PI3K, p-PI3K, AKT, p-AKT, STAT3, p-STAT3 were purchased from Cell Signaling Technology, β-Actin was purchased from Santa Cruz Biotechnology. The secondary antibodies were purchased from Odyssey.

### MTT Assay

A549 cells and PC-9 cells were seeded in 96-well plates and cultured overnight of adhesion, then treated with different concentrations of honokiol (0, 20, 40, 60, and 80 μM) for 24, 48, and 72 h, respectively; 10 μl of MTT solution (5 mg/ml) was added in each well and incubated for another 4 h. Then 100 μl of DMSO was added in each well and incubated for 4 h to dissolve the formazan crystals. Absorbance of plates was measured at 570 nm with Tecan microplate reader (Morrisville, NC, United States).

### Colony Formation Assay

PC-9 cells were seeded in dishes with a diameter of 60 mm with 500 cells/dish and cultured overnight of adhesion, then treated with different concentrations of honokiol (0, 20, 40, 60, and 80 μM) with medium changes per 3 days until visible colonies formed. The colonies were washed by PBS and fixed with 4% paraformaldehyde and stained with Wright-Giemsa stain. The number of colonies formation in each dish was counted.

### Wound Healing Assay

PC-9 cells were seeded in 6-well plates with the concentration of 2 × 10^5^ cells/ml. Scratch wounds were made by scraping the cell layer with the tip of 10 μl pipette, debris was removed by washing the cells with 1 × PBS, then three fields (40×) were randomly picked from scratch wound of each well. After wounding, cells were exposed to various concentration of honokiol (0, 20, 40, 60, and 80 μM) for 12 and 24 h, three random fields (40×) were picked from scratch wound at each exposed time.

### Transwell Invasion Assay

Transwell membranes (pore size: 8 μm) coated with Matrigel (BD Biosciences, United States) were re-hydrated for 1h in an environment of 37°C in FBS-free RPMI-1640 medium. PC-9 cells were resuspended into FBS-free RPMI-1640 medium with various concentration of honokiol (0, 20, 40, 60, and 80 μM) and seeded into the upper chamber at a density of 5 × 10^5^ cells/ml. 600 μl RPMI-1640 medium with 10% FBS was added into the lower chamber. After 24 h incubation, Transwell membranes were with 4% paraformaldehyde for 30 min and then stained with Wright-Giemsa stain. Non-invading cells on the upper surface of the membrane were removed. Five randomly fields were picked from every membrane with microscope at 400× magnification.

### Apoptosis Assay

PC-9 cells were seeded in 6-well plates and exposed to various concentration of honokiol (0, 20, 40, 60, and 80 μM) for 24 h. Annexin V-FITC solution and PI solution were used to stain cells in the dark for 15 min. Each sample was analyzed by flow cytometry and the percentages of apoptotic cells of every group were analyzed with Flow J software.

### Western Blots Analysis

Cells were lysed in RIPA lysis buffer and kept in ice for 30 min. Then the lysate was centrifuged at 4°C, 12000 rpm for 10 min. 20 μg of each protein samples were loaded into the lane of 10% SDS-PAGE gel with two lane of 2 μl protein molecular weight marker for separation, then transferred the protein to PVDF membrane. Non-specific binding was blocked with 5% no-fat milk which diluted in 1 × TBST for 1 h and washed three times with 1 × TBST. The membranes were incubated with primary antibodies (1:1000) at 4°C overnight. After removed the extra primary antibodies and washed three times with 1 × TBST, the membranes were incubated with secondary antibody (1:1000) for 1 h at room temperature. The bands were visualized by the Pierce ECL Western Blotting Kit or LI-COR Odyssey Scanner.

### Cell Transfection

For Lyn knockdown, PC-9 cells were seeded in 6-well plates. When the cells reached 80% confluence, the medium was replaced with FBS-free RPMI1640 medium and cells were transfected with Lyn siRNA and Lipofectamine 2000. The Lyn expression was analyzed by Western blots.

### Statistical Analysis

All of the statistical analyses were conducted by the SPSS 17.0 software and all the data was expressed as Mean ± SEM. Statistical significance differences were evaluated by one-way ANOVA and using LSD or Tamhane’s method for comparison tests between two groups. The level of statistical significance was defined as *P* < 0.05.

## Author Contributions

X-JY, G-PL, and EL: conceived and designed the study. XD, R-ZL, Z-BJ, C-LW, and L-XL: performed the experiments. XD and EL: wrote the paper. All authors read and approved the final manuscript.

## Conflict of Interest Statement

The authors declare that the research was conducted in the absence of any commercial or financial relationships that could be construed as a potential conflict of interest. The reviewer PL declared a shared affiliation, with no collaboration, with the authors to the handling Editor.
